# CuO and CeO_2_ Nanostructures Green Synthesized Using Olive Leaf Extract Inhibits the Growth of Highly Virulent Multidrug Resistant Bacteria

**DOI:** 10.3389/fphar.2018.00987

**Published:** 2018-09-07

**Authors:** Qaisar Maqbool, Mudassar Nazar, Ayesha Maqbool, Muhammad T. Pervez, Nyla Jabeen, Talib Hussain, Gregory Franklin

**Affiliations:** ^1^Department of Integrative Plant Biology, Institute of Plant Genetics of the Polish Academy of Sciences, Poznan, Poland; ^2^Department of Biotechnology, Virtual University of Pakistan, Lahore, Pakistan; ^3^National Institute of Vacuum Science and Technology, Islamabad, Pakistan; ^4^Department of Molecular Biology, Virtual University of Pakistan, Lahore, Pakistan; ^5^Department of Bioinformatics and Computational Biology, Virtual University of Pakistan, Lahore, Pakistan; ^6^Applied Biotechnology and Genetic Engineering Lab, Department of Bioinformatics and Biotechnology, International Islamic University, Islamabad, Islamabad, Pakistan

**Keywords:** green synthesis, CuO-nanostructures, CeO_2_-nanostructures, multidrug-resistant bacteria, cytotoxicity, biocompatibility

## Abstract

One of the major challenges of nano-biotechnology is to engineer potent antimicrobial nanostructures (NS) with high biocompatibility. Keeping this in view, we have performed aqueous olive leaf extract mediated one pot facile synthesis of CuO-NS and CeO_2_-NS. Prepared NS were homogenous, less than 26 nm in size, and small crystallite units as revealed by scanning electron microscopy (SEM) and X-ray diffraction (XRD) analyses. Fourier transform infrared spectroscopy (FTIR) of CuO-NS and CeO_2_-NS showed typical Cu-O prints around 592–660 cm^-1^ and Ce-O bond vibrations at 453 cm^-1^. The successful capping of CuO-NS and CeO_2_-NS by compounds present in the plant extract was further validated by high performance liquid chromatography (HPLC) and thermal gravimetric analysis (TGA). Active phyto-chemicals from the leaf extract simultaneously acted as strong reducing as well as capping agent in the NS synthesis. NS engineered in the present study showed antibacterial potential at extremely low concentration against highly virulent multidrug-resistant (MDR) gram-negative strains (*Escherichia coli*, *Enterobacter cloacae*, *Acinetobacter baumannii* and *Pseudomonas aeruginosa*), alarmed by World Health Organization (WHO). Furthermore, CuO-NS and CeO_2_-NS did not show any cytotoxicity on HEK-293 cell lines and Brine shrimp larvae indicating that the NS green synthesized in the present study are biocompatible.

## Introduction

Bacterial epidemiology, microbial invasions, drug resistance, and random mutations are the hot topics under discussion today. There is a race between drug development and bacterial resistance (Puzyn et al., 2011; Saravanakumar et al., 2017). The loss of efficiency to cure microbial infections is persistently observed for several drugs (Puzyn et al., 2011). Many antimicrobial agents that revolutionized treatment against infections in the past have now lost their bactericidal capabilities (Zaman et al., 2017). The potential threat to mankind gets higher when WHO issued the list of multi-drug-resistant (MDR) pathogen in 2017, which includes *Enterobacteriaceae*, *Acinetobacter*, and *Pseudomonas*. According to WHO observations, these bacteria are resistant even to the strongest third generation antibiotics (cephalosporin group). It is strongly predicted that death toll due to drug resistant pathogens may rise up (Rather et al., 2017; Zaman et al., 2017; Grzelak et al., 2018).

Due to multiple modes of action, nanostructures (NS) have been successfully used against MDR bacterial pathogens. The ability to fine-tune the morphological, optical, magnetic, and physical properties of metal oxide NS makes them suitable agents for biomedical and biotechnological applications (Wang X. et al., 2016; Caballero-Calero and D’Agosta, 2017). Due to extremely small size and high reactivity, these NS could target the surface envelop and even the genomic content of bacterial pathogens. Maximum penetration of the bacterial cell wall by NS has been observed due to opposite charges of attraction. These unique properties of multimode of actions and maximum invasion are quite helpful in developing NS as broad-spectrum antibiotics in the future (Maqbool et al., 2017; Ni et al., 2017).

Among metal oxide NS experimented so far, the performance of CuO-NS and CeO_2_-NS was found extremely effective in biological applications (Anwaar et al., 2016). CeO_2_-NS exhibits variable oxidation states, stable crystal structure, greater surface energy, high surface to charge ratio, visible light activation, and greater stability making it as an ideal candidate for biomedical applications (Charbgoo et al., 2017; Kamila and Venugopal, 2017; Chen and Stephen Inbaraj, 2018). All these characteristics are directly linked to variable oxidation states of Ce (Ce^3+^, Ce^4+^) and photoexcitaion at room temperature through which the NS can generate lethal reactive oxygen species (ROS) (Maria Magdalane et al., 2017). When tested against lethal strains like *Escherichia coli*, *Staphylococcus aureus*, and *Pseudomonas aeruginosa*, CuO-NS showed moderate antibacterial behavior (Maqbool et al., 2017).

Although a variety of metal oxide NS have been tested for advanced biomedical applications, the extensive use of synthetic reagents during their chemical synthesis makes these NS least biocompatible. Green synthesis of NS using plant extract has gained a lot of importance because of the bio-safety and economy of NS prepared by this method. Olive leaf aqueous extract contains a variety of phyto-reductants for tailoring NS. The biomedical potential of olive is well known primarily due to the presence of antioxidants like oleuropein, oleuroside and apigenin-7-O-glucoside (Lim et al., 2016; Maalej et al., 2017; Marslin et al., 2018).

In this study, we report on the comparative analysis of green synthesized CuO-NS and CeO_2_-NS for their biocompatibility, cytotoxicity and most importantly antimicrobial potential. Results presented here will help us to understand the performance of green synthesized CuO-NS and CeO_2_-NS in future biomedical applications.

## Materials and Methods

### Green Synthesis of CuO-NS and CeO_2_-NS Using Olive Leaf Extract

Olive leaves (*Olea europaea*) were collected and washed three times with ddH_2_O. To avoid any damage to light sensitive bioactive compounds, collected leaves were dried under shade. Later on, they were ground in to fine powder. To prepare the extract, 30 g of leaf powder was added to an Erlenmeyer flask containing 300 mL of ddH_2_O and shaken at 50 rpm at 50°C in an incubator. After 2 h, the mixture was filtered through a Whatmann No. 1 filter paper and the filtrate was stored in a refrigerator at 15°C.

For the green synthesis of CeO_2_-NS, 13.02 g of (CeNO_3_)_3_. 6H_2_O was added to 300 mL of plant extract in an Erlenmeyer flask. The reaction mixture was stirred at 1,500 rpm at 50°C on a magnetic plate. After 2.5 h of stirring, the reaction mixture was centrifuged at 10,000 rpm (GR Bio-Tek centrifuge, Orpington, England) for 10 min to pellet the synthesized CeO_2_-NS. Dark brown color CeO_2_-NS pellets were obtained. The pellets were washed three times with ddH_2_O. In the next step, all of the washed CeO_2_-NS pellets were placed in Hot-Air-Oven setup to 60°C for 6.5 h. In order to achieve greater crystallinity, CeO_2_-NS were further calcined inside a Gallenkamp furnace (Apeldoorn, Netherlands) at 500°C for 2.5 h. A similar procedure was adopted for CuO-NS synthesis by using 5.43 g of Cu(CO_2_CH_3_)_3_ in 300 mL of olive leaf extract. Prepared NS were stored in airtight containers under ambient conditions. The step-by-step process of facile green synthesis of CuO-NS and CeO_2_-NS is illustrated in **Figure 1**.

**FIGURE 1:** Scheme showingfacile green synthesis of NS using olive leaf extract.

### High Performance Liquid Chromatography (HPLC) Analysis of Plant Extract

For the identification of active bio-molecules present in the olive leaf extract used in the green synthesis, it was subjected to HPLC analysis as described before (Miller, 2017). Briefly, 5 g of olive leaf powder was added to 30 mL of aqueous methanol (60%) and thoroughly mixed in a blender. The resulting mixture was centrifuged at 3,000 rpm for 5 min. The supernatant was collected and filtered through 0.22 μm micro-filter. Separation of compounds was performed in an HPLC (Agilent 1100 Technologies, Ireland) using water-acetic acid (99.5–0.5) as mobile phase-A and acetonitrile as mobile phase-B. The flow rate of the column was set at 1 mL/min along with temperature set at 25°C. Compounds were examined based on retention time (t_R_) and elution time (t_o_) for unretained peak. Moreover, polyphenolic compounds from olive extract were identified using two systems of liquid chromatography hyphenated to mass spectrometers following the method of Piasecka et al. (2015). The first system consisted of HPLC Agilent 1100 coupled to Esquire 3000 (Bruker Daltonics) ion trap mass spectrometer and the second was UPLC (Acquity Waters) hyphenated to QExactive hybrid MS/MS quadrupole-Orbitrap instrument (Thermo). Compounds were identified according to exact masse of their [M+H]+ and [M-H]- ions; their fragmentation patterns and chromatographic retention times by comparison with standard compounds (Sigma-Aldrich).

### Characterization of CuO-NS and CeO_2_-NS

#### Thermal Gravimetric Analysis (TGA) of CuO-NS and CeO_2_-NS

The thermal stability and bio-molecular capping action around green synthesized NS were evaluated using PerkinElmer-Diamond-TGA (Llantrisant, United Kingdom). The temperature increment was set between 25.00 and 800.00°C with increase of 10.00°C/min.

#### Fourier Transform Infrared Spectroscopy (FTIR) of CuO-NS and CeO_2_-NS

Vibrational bond energies and molecular nature of NS were examined by FTIR spectroscopy (SHIMADZU FTIR) with wave number set between 400 and 4,000 cm^-1^ following KBr pellet method.

#### X-ray Diffraction (XRD) Analysis

Crystallographic parameters of green synthesized NS were checked with PANalyticalX′Pert^3^ powder machine (Royston, United Kingdom) powered with Ni-Monochromator, and machine diffraction angel (2𝜃) specific for crystalline materials (20–80°). In XRD analysis, Cu_Kα radiation of specific wavelength 1.5406 Å was used. In order to determine the crystallite size value of bio-fabricated NS, Scherer’s equation [*D* = 0.9λ/βcos𝜃] was applied. From the values of equation, D is the average crystalline domain size perpendicular to the reflecting planes, λ is showing the X-ray wavelength (1.5406 Å), ß is the angular full width at half maximum (FWHM) in radians and 𝜃 is the diffraction angle [2𝜃 (degree) is the calculated angle of diffraction in degree] or also known as Bragg’s angle.

#### Scanning Electron Microscopy (SEM) of CuO-NS and CeO_2_-NS

Measurement of NS size and surface morphology is important for NS based biological applications. Hence, the size and surface structure of fabricated CuO-NS and CeO_2_-NS were analyzed using JOEL-JSM-6490LA-SEM (Tokyo, Japan) setup at 20 kV with counting-rate of 2838.

### Antibacterial Activity of CuO-NS and CeO_2_-NS

To screen the antibacterial potential of CuO-NS and CeO_2_-NS, *E. coli* (ATCC 25922), *E. cloacae* (ATCC 23373), *A. baumanni* (ATCC 19606), and *P*. *aeruginosa (ATCC* 27853) strains were tested via disc diffusion method as we reported before (Maqbool et al., 2016). In detail, bacterial strains were cultured in nutrient broth culture (Sigma-Aldrich) at 37°C until reaching 1.5 × 10^8^ colony forming unit (CFU) per mL. Bacteria were carefully spread on Petri dishes containing semi-solid culture medium. Sterilized filter paper discs loaded with 5 μL solution containing 20 μg/μL of NS. Discs loaded with 5 μL roxithromycin (4 mg/mL) were considered as positive control, while discs loaded with deionized H_2_O was used as negative control. All of the inoculated plates were placed in the incubator set for 37°C and the zone of inhibition (ZOI) was measured after 24 h.

### Cytotoxicity Assay of Green Synthesized CuO-NS and CeO_2_-NS on HEK-293 Cells

Cell viability assay was performed following the method as described previously (Abbas et al., 2017a). HEK-293 cells (Sigma-Aldrich) were seeded in a 96-well plate at a concentration of 10^5^ cells per well and incubated at 37°C under 5% CO_2_ environment to allow cell adhesion. After 24 h of incubation, the wells were added with different concentrations of the CuO-NS and CeO_2_-NS (0.01, 0.05, and 0.1 mg/mL). The cell viability was examined via CCK-8 analyzer and OD was recorded at 450 nm by Multi Scan MK3 after 24 h of NS treatment.

### Examination of Biocompatibility of Green Synthesized CuO-NS and CeO_2_-NS (Using Brine Shrimp Larvae)

The biocompatibility of green synthesized CuO-NS and CeO_2_NS was tested via Brine shrimp (*Artimia salina*) lethality assay. Brine shrimp eggs procured from Ocean-Star-International (Coral Springs, United States). They were maintained in 3.8% (w/v) saline water (Coral Springs, United States) at 37°C for 2 days for hatching. 48 h after hatching, the larvae were collected using Pasteur pipette. To each vial containing different concentrations (5, 10, and 15 mg/mL) of CuO-NS and CeO_2_NS in saline water was transferred with 10 larvae. Larvae transferred to vials containing doxorubicin dissolved saline water (10 μg/mL*)* and to vials containing only saline water served as negative and positive controls, respectively. All the vials with larvae were incubated at 28°C. After 24 h of incubation, the number of live and dead larvae was counted manually with the aid of a magnifying glass to calculate the LD_50_ value of NS.

### Statistical Analysis

All the experiments were repeated at least three times and the values are presented as the mean ± SD. Statistical investigation of the results was done by student’s *t*-tests using SPSS software. *P* < 0.05 considered significant.

## Results

### HPLC and TGA Findings

HPLC analysis of olive leaf extract revealed the presence of several secondary metabolites (**Figure 2**). They were oleuroside (*t_R_* = 33.8), oleuropein (*t_R_* = 23.6), isoquercetin (*t_R_* = 12.5), apigenin-7-O-glucoside (*t_R_* = 16.2), luteolin-7-glucoside (*t_R_* = 8.9), verbascoside (*t_R_* = 7.9), rutin (*t_R_* = 6.7), and hydroxytyrosol (*t_R_* = 2.5).

**FIGURE 2:** HPLC chromatogram showing major compounds present in the olive leaf extract **(top)** with hypothesized capping action around NS **(bottom)**.

Capping action around CuO-NS and CeO_2_-NS was evaluated through TGA analysis. When the green synthesized NS were subjected to progressively increasing temperature, the loss of weight in NS was observed in three phases. In the first phase from 50 to 100°C, the loss of weight was due to surface absorbed H_2_O. In the second phase from 100 to 200°C, there was the breakdown of capping agent, which resulted in combustion of capping agent attached to the surface of NS, which might be connected with oleuropein originated organic compound (C_8_H_10_O_3_). The thermal decomposition of CuO-NS and CeO_2_-NS observed in the third phase at 600°C was due to high temperature oxygen decay. TGA findings are shown in **Figure 3**.

**FIGURE 3:** Graphical presentation of thermal gravimetric analysis (TGA) of the green fabricated NS showing the progressive decomposition of capping agent with increasing temperature.

## Characterization of CuO-NS and CeO_2_-NS

### FTIR Studies of Green Synthesized CuO-NS and CeO_2_-NS

FTIR analysis revealed the successful reduction of precursor ionic complexes of CuO-NS and CeO_2_-NS in **Figure 4**. The reading around 2,800 cm^-1^ represents the presence of surface adsorbed H-O-H molecules. The vibration modes from 2,500 to 4,000 cm^-1^ are showing C-O, O-H and H-H bond order frequencies. Cu-O identification peaks were traced at 592, 607, and 665 cm^-1^. While Ce-O stretching bond frequencies were found at 453 cm^-1^.

**FIGURE 4:** FTIR spectra of CuO-NS and CeO_2_-NS green-synthesized using olive leaf extract.

### XRD Studies of CuO-NS and CeO_2_-NS

XRD results are important to predict the crystallite size, crystal shape, grain boundaries, phase purity, doping results, and total surface area of engineered NS. **Figure 5** represents the typical XRD spectrum of CuO-NS and CeO_2_-NS prepared after calcination. Both of the samples reflect absolute pure crystalline phase with no additional peaks indicating that there are no other impurities. In case of CuO-NS, all of the Braggs peaks are well corresponding to JCPDS-05-0661 (Card-No.), while the Braggs peaks of CeO_2_-NS are similar to JCPDS-340394 (Card No.). This similarity index clearly indicates the pure crystalline morphology of green synthesized NS. CuO-NS crystallite size calibrated through Scherer approximation is 5 nm while CeO_2_-NS crystallite size is found 6 nm. Crystallographic design validates that each Ce atom in a crystallite is surrounded by eight oxygen atoms showing face-centered cubic geometry.

**FIGURE 5:** XRD analysis of prepared CuO-NS and CeO_2_-NS.

### SEM Analysis of Green Synthesized CuO-NS and CeO_2_-NS

As revealed by the SEM imaging (**Figure 6**), all the prepared NS were spherical and highly homogenous and the average size of CuO-NS and CeO_2_-NS was 22 ± 02 and 24 ± 04 nm, respectively.

**FIGURE 6:** SEM images of **(A)** CuO-NS **(B)** CeO_2_-NS.

### Antibacterial Activity of Green-Synthesized CuO-NS and CeO_2_-NS

**Figure 7** shows the ZOI exhibited by CuO-NS and CeO_2_-NS treatment against the tested MDR pathogens. All the strains were successfully inhibited by both CuO-NS and CeO_2_-NS. The maximum ZOI against *E. coli* was 18.3 mm and 21.2 mm, respectively, for CuO-NS and CeO_2_-NS. Moreover, due to the divergent physio-chemical characteristics of Cu and Ce, both of them have shown differential inhibitory behavior. Olive leaf extract has also shown mild inhibitory action with maximum ZOI of 8 mm against *E. cloacae*.

**FIGURE 7:** Graph showing the zone of inhibition recorded for various MDR pathogens against CuO-NS, CeO_2_-NS, plant extract, roxithromycin (positive control) and deionized water (negative control).

### Cytotoxicity and Biocompatibility Testing of Green Synthesized CuO-NS and CeO_2_-NS on HEK-293 Cells and Brine Shrimp Larvae

**Figure 8** represents the effect of different concentrations (0.01, 0.05, and 0.1 mg/mL) of CuO-NS and CeO_2_-NS on HEK-293 cell lines. It is quite obvious from the findings that both of the NS show no or mild cytotoxicity to the HEK-293 cells even at relatively high concentration of 0.1 mg/mL. Mild cytotoxicity was observed for green synthesized NS at very high concentration of 0.05 mg/mL.

**FIGURE 8:** Effect of green synthesized NS on HEK-293 cell viability.

We have selected Brine shrimps, as their early developmental stages are very sensitive to toxic agents, and the toxicity symptoms could be easily observed. Biocompatibility assay with Brine shrimps larvae shows that both CuO-NS and CeO_2_-NS are non-toxic to them up to 10 mg/mL. When increasing the concentration of to 15 mg/mL, CuO-NS and CeO_2_-NS caused 20 and 30% mortality, respectively (**Table 1**). At this concentration, 100% mortality of larvae was observed in doxorubicin treatment.

**Table 1:** Analysis of CuO-NS and CeO_2_-NS, toxicity to Brine shrimp larvae.

Sample	Different concentration of NS applied								
	5 mg/mL			10 mg/mL			15 mg/mL		
	
	T	L	% M	T	L	% M	T	L	% M
CuO-NS	10	10	00	10	09	10	10	08	20
CeO_2_-NS	10	10	00	10	08	20	10	07	30
*Olive* extract	10	10	00	10	10	00	10	10	00
(Negative) control	10	10	00	10	10	00	10	10	00
Doxorubicin (positive control)	10	01	90	10	06	40	10	00	100

*T, no. of A. salina added; L, alive A. salina after 24 h; %M, % mortality.*

## Discussion

### Role of Phyto-Reductants and Capping Agents for Tailoring CuO-NS and CeO_2_-NS

The abundance of oleuropein over other phenolic compounds was observed in HPLC chromatogram of olive leaf extract (**Figure 2**), as reported in previous studies (Lim et al., 2016; Maalej et al., 2017). Oleuropein is highly unstable molecule and will rapidly breakdown into more polarizable hydroxytyrosol (C_8_H_10_O_3_) usually in organic solvents (Maqbool et al., 2016). This molecule might have been involved in the capping action around high-energy planes (atoms) in tailoring CuO-NS and CeO_2_-NS in the present study. It could simultaneously act as phyto-reducing and phyto-capping agent during the NS synthesis. TGA findings (**Figure 3**) supplement the HPLC observations. When the green synthesized NS were subjected to increasingly high temperature, there was a breakdown of surface capping agent (hydroxytyrosol), which resulted in the combustion of bio-capping agent attached to the surface of NS. The thermal decomposition of CuO-NS and CeO_2_-NS around at 600°C was due to high temperature oxygen decay (El-Nahhal et al., 2016; Maqbool, 2017).

### Characterization of Green-Synthesized CuO-NS and CeO_2_-NS

FTIR was used to analyze the chemical composition and surface chemical coordinates of the CuO-NS and CeO_2_-NS (**Figure 4**). The vibration modes from 2,500 to 4,000 cm^-1^ are showing C-O, O-H, and H-H bond order frequencies (Maqbool et al., 2016; Maqbool, 2017). Cu-O identification peaks were traced at 592, 607, and 665 cm^-1^. While Ce-O stretching bond frequencies were found at 453 cm^-1^. Corresponding findings related to Cu-O and Ce-O are well indexed to previously reported studies (Zayyoun et al., 2016; Maqbool, 2017).

Crystallite size, crystal shape, grain boundaries, phase purity, doping results, and total surface area of engineered NS are important factors for antibacterial performance. Smaller crystallite size will provide greater penetration capabilities with maximum absorption rate (Adhikari et al., 2018). Smaller will be the crystallite size, greater will be the value of quantum confinement effect, which is responsible for the overall reactivity and surface activation of the electron during the reaction (Thanh et al., 2014). NS synthesized in the present study possess ideal reduction in crystallite size (see **Figure 5**) with an overall homogenous morphology which augmented greater reactivity to their structure for antimicrobial applications.

Since the size and shape of NS will define their reactivity, surface area, rate of absorption into microbial cell, cell surface interaction, protein binding etc. (Adhikari et al., 2018), these parameters are of prime importance for antimicrobial applications. SEM findings as presented in **Figure 6** supports green synthesized CuO-NS and CeO_2_-NS behavior for greater penetration to tissue.

### Antibacterial Potential of Green-Synthesized CuO-NS and CeO_2_-NS

Due to the divergent physio-chemical characteristics of Cu and Ce, both of them have shown differential inhibitory behavior. Phyto-reductants from olive leaf extract have also shown mild inhibitory actions and these bactericidal properties of olive plant extract are well known in literature (Lim et al., 2016; Maalej et al., 2017).

The observed difference in the ZOI between bacterial strains may be due to unique bacterial cell wall morphology that assists pathogens to oppose against applied antimicrobial NS. In addition to this, other characteristics like the rate of NS diffusion across bacterial envelop, chemical properties, binding activation energy, ionic discharge and surface charge attraction also play the key role against a range of bacterial pathogens (Lu et al., 2017; Wang L. et al., 2017). Gram negative pathogens also possess structural differences in cell wall like the deposition of lipopolysaccharide material which augments more virulence to them. Furthermore, it has been commonly observed that green synthesized NS own low level of genotoxic and cytotoxic nature for normal somatic cells with proven efficiency as compare to NS produced by other physical or chemical methods (Devipriya and Roopan, 2017; Lu et al., 2017). Doped or undoped CeO_2_-NS engineered by various chemical procedures also showed cytotoxicity to healthy cells (Abbas et al., 2017a; Dekkers et al., 2017).

Current findings explore that green-synthesized NS are of extremely small size, homogenous morphology, smaller crystallite size, enhanced surface area, and are of pure chemical nature. All these properties cumulatively contributed toward supreme antibacterial action. Smaller size and positively charged NS can easily be attracted by negatively charged bacterial surface. This electrostatic force of attraction is quite helpful in auto-phagocytosis of NS inside the bacterial cellular environment (Maqbool et al., 2016, 2017). Normally, it has been observed that due to the presence of additional mucus layer (lipopolysaccharide), it is a tough task for any drug molecule to penetrate across it. But due to the optimized charged surface, NS probably can penetrate through cellular covering. In some of the previously observed bactericidal activities, thiol (-SH) group present in the bacterial cell surface protein also have shown strong affection for metal oxide NS, due to which NS may also involve in denaturation of bacterial surface proteins (El-Nahhal et al., 2016; Lu et al., 2017).

Cu possesses variable oxidation state between Cu^+^ and Cu^2+^. This is primarily because most of the transition metals can involve either 3 d or 4 s shells for electron shuffling (Wang S. et al., 2017). It is commonly observed that variable oxidation states of metal ions can produce lethal ROS when exposed to the cellular environment. Ce also own variable oxidation state of Ce^3+^ and Ce^4+^, which also supports ROS burst and activation of redox process during antibacterial action (Charbgoo et al., 2017). Metal ions from NS are even more reactive and highly responsible for ROS generation. In our study, the antibacterial activity might also be strongly linked to the photo-activation of ROS by NS on bacterial growth as hypothesized in **Figure 9**. Lethal ROS species (OH^-^, _1_O^2-^, ^∗^O_2_) interact with the cellular environment and produce greater oxidative stress. Increase in oxidative stress causes direct genome destruction, plasmid and cell protein denaturation, ROS-induced mitochondrial damage and partial or absolute loss of cell wall permeability (Li et al., 2016; Kung et al., 2017). The multimode of actions performed by green fabricated CuO-NS and CeO_2_-NS causes complete growth inhibition of all of the MDR bacterial strains.

**FIGURE 9:** Biocompatibility of green synthesized NS (ROS generation in bacterial cell causes lethal effects, while NS applied on Brine Shrimp are shown non-toxic).

### Bio-Compatibility Testing of Green Synthesized CuO-NS and CeO_2_-NS on HEK-293 Cells and Brine Shrimp Larvae

It is very important that while targeting the pathogen, NS must not harm the somatic cell environment. NS synthesized from the physical or chemical methods are found toxic to healthy cells (Asharani et al., 2008). This is probably due to the extensive use of hazardous acid base synthetic reagents in NS preparation by these methods (Dekkers et al., 2017). On the other hand, green chemistry proves to be an efficient and most reliable method to engineer highly biocompatible NS (Abbas et al., 2017b). Moreover, mild cytotoxicity activities of green-synthesized NS are probably due to high concentration metal ion intoleration, NS sedimentation, loss of NS-homeostasis, genotoxicity, or lethal ROS induction (Li et al., 2016). Overall testing concludes that CuO-NS and CeO_2_-NS are differentially cytotoxic toward gram-negative bacteria as compared to normal body cells.

Cytotoxic assay (**Table 1**) evidently demonstrated that both CuO-NS and CeO_2_-NS are not toxic to Brine shrimp larvae. In order to achieve efficient drug development, it is vital to have the understanding of the toxicity of synthesized NS. Normally it has been observed that metal oxide NS show differential cytotoxicity when applied on healthy cells (Abbas et al., 2016). In the current study, olive leaf extract mediated synthesis of NS demonstrates greater biocompatibility with the least lethal effect on Brine shrimps larvae as shown in **Figure 9**. Even at higher dosage, minor lethality was reported. This mild lethal effect shown by CeO_2_-NS (30% with 15 mg/mL) is probably due to sedimentation of heavy Ce-metal ions, alteration in cellular metabolism and lethal ROS production (Gliga et al., 2017).

## Conclusion

We have successfully fabricated the CuO-NS and CeO_2_-NS using bio-reductants from olive leaf extract and have achieved the following outcomes:

• HPLC analysis of plant extract and TGA findings of CuO-NS and CeO_2_-NS confirms the successful capping action performed by phytochemicals around NS. The NS are of extremely small size (SEM results) and homogenous.
• XRD findings validate the pure chemistry of green-synthesized CuO-NS and CeO_2_-NS with small crystallite size.
• FTIR spectrum demonstrates single phase and pure chemical nature of chemically bonded Cu-O and Ce-O in prepared CuO-NS and CeO_2_-NS, respectively.
• Although the green fabricated CuO-NS and CeO_2_-NS could completely inhibit the growth of MDR bacterial strains, they are not toxic to healthy HEK-293 cells and Brine shrimp larvae.

So, green synthesis proves to be the most reliable method for achieving biocompatible NS. We believe that NS reported in the present study might have the potential to fight against antibiotic resistant pathogenic bacteria in the near future.

## Author Contributions

QM and MN contributed to major part of the research work. GF provided his expert opinion and technical expertise related to the accomplishment of biomedical application part. The remaining authors contributed equally.

## Conflict of Interest Statement

The authors declare that the research was conducted in the absence of any commercial or financial relationships that could be construed as a potential conflict of interest.
